# Next-Day Medical Activities Recommendation Model with Double Attention Mechanism Using Generative Adversarial Network

**DOI:** 10.1155/2022/6334435

**Published:** 2022-11-07

**Authors:** Wei Li, Jinzhao Yang, Xin Min

**Affiliations:** ^1^Key Laboratory of Intelligent Computing in Medical Image (MIIC), Northeastern University, Ministry of Education, Shenyang 110000, Liaoning, China; ^2^School of Computer Science and Engineering, Northeastern University, Shenyang 110000, Liaoning, China

## Abstract

Medical activities recommendation is a key aspect of an intelligent healthcare system, which can assist doctors with little clinical experience in clinical decision making. Medical activities recommendation can be seen as a kind of temporal set prediction. Previous studies about them are based on Recurrent Neural Network (RNN), which does not incorporate personalized medical history or differentiate between the impact of medical activities. To address the above-given issues, this paper proposes a Next-Day Medical Activities Recommendation (NDMARec) model. Specifically, our model firstly proposes an inpatient day embedding method based on soft-attention which balances the impact of different medical activities to get a joint representation of medical activities that occurred within the same day. Then, a fusion module is designed to combine features of inpatient day and medical history to achieve personalization. These features are learned by the self-attention mechanism that solves the long-term dependency problem of RNNs. Last, adversarial training is introduced to improve the generalization ability of our model. Extensive experiments on a real dataset from a hospital are conducted to show that NDMARec outperformed both classical and state-of-the-art methods.

## 1. Introduction

As populations grow and societies develop, the demand for high-quality healthcare services continues to rise, while regional and national differences in healthcare quality continue to become greater. Young physicians who lack clinical experience have difficulty making effective clinical decisions when faced with unfamiliar conditions. In addition, public health emergencies, such as the COVID-19 outbreak, have had a dramatic impact on the healthcare system. In recent years, artificial intelligence (AI) has shown great potential for development. Therefore, if AI technology can be effectively used to achieve accurate recommendations for clinical medical activities, the overall quality of healthcare services will be greatly improved. The motivation for this work is to train recommendation models to assist young physicians who lack clinical experience with related diseases to make effective clinical decisions in the face of unfamiliar diseases. It helps inexperienced physicians to plan followup treatment by recommending next-day medical activities.

Previous research on Electronic Medical Record (EMR) mostly focused on risk prediction [1] and readmission prediction [2]. In recent years, related researches are more focused on the prediction of the next clinical event [3]. The difficulty they encounter is how to weigh the accuracy of the results against the intelligibility. Neural network models usually have higher accuracy than simple statistical models but are not as intelligibile. Next-day medical activities recommendation does not simply predict a clinical event but recommend a set containing multiple medical activities, which can be seen as a special next-basket recommendation [4] or temporal set prediction [5]. The difficulty of the temporal set prediction problem is how to efficiently represent a set and capture the temporal relationships between different sets. Next-day medical activities recommendation models likewise need to have good comprehensibility, which is the key to medical application models. And, the difficulty of the temporal set prediction problem is also present in our study. Thus, It is still a challenging task in the medical domain.

Firstly, it is difficult to achieve an effective representation of the medical activity set. What it intends to denote is related to the medical activities that occurred on that day, but the importance of the medical activities is different. For example, a patient takes vitamin B12 and capecitabine (a chemotherapy drug) on a given day. Obviously, the latter is more important. Hence, it is a challenge to highlight information on important medical activities without losing information on ancillary medical activities when generating inpatient day embedding. Secondly, the relationship between inpatient days is difficult to describe, which includes both chronological and causal relationships. For example, a patient is allergic to a particular medication that is first tried, so a new medication is switched to the next-day's medical activity. Thirdly, when doctors formulate medical activities for inpatients, they are influenced by the earlier medical history in addition to the current condition. All the independent recommendation model learns about is the treatment pattern between inpatient days, but the individual features of inpatients are not emphasized. Inspired by [6], a generative adversarial network is used to solve this problem. The goal is to train the recommendation network to learn effective features which can recommend medical activities which better match the individual characteristics of inpatients. The discriminator specifically distinguishes between machine-recommended medical activities and real next-day medical activities and is used as an adversary for the recommendation network. If the discriminator is able to distinguish between the recommended medical activities and the real medical activities, the recommendation network is penalized.

Here, the recommended medical activities we considered should be more in line with the real distribution of next-day medical activities. Firstly, the recommended set of medical activities should include the actual set of next-day medical activities as much as possible. Secondly, the elements in the intersection of the two sets should be ranked as high as possible in the recommended set of medical activities, i.e., the corresponding recommendation score should be as high as possible. Finally, the recommended medical activities are personalized as much as possible, rather than generic medical activities such as general food and nursing care.

To solve the above-given issues, we propose a new attention-based neural network for next-day medical activities recommendation, which consists of four components: inpatient day embedding, multihead self-attention mechanism, information fusion, and generative adversarial networks. A soft-attention mechanism is used to generate inpatient day embedding to balance the impact of different medical activities. Potential relationships within inpatient day sequences and word features of medical history are extracted by multihead self-attention to alleviate long-term dependency and enable parallel computing. Medical activity and historical information are fused, which allows personalized information about the inpatient to be added when recommending the next-day medical activities. A generative adversarial network is used in the model training stage to improve the generalization ability of the recommendation network.

The contributions of this paper can be summarized as follows:

- A novel recommendation model for next-day medical activities is proposed, which considers the personalized impact of medical history and the importance of different medical activities and formalize them as attention factors.
- Generative Adversarial Network is used to improve the quality of recommendations, which enforces the network to learn features which can be used to recommend activities with a distribution which resembles activities that occurred really.
- Extensive experiments on a real dataset from a top-notch hospital validate the superiority and interpretability of NDMARec.

The rest of this paper is organized as follows: Section 2 reviews previous work related to the problem studied in this paper.  Section 3 presents the formalization of the problem.  Section 4 describes in detail each component proposed by our framework and model.  Section 5 evaluates the proposed approach through experiments. Finally, Section 6 concludes the whole paper.

## 2. Related Work

### 2.1. Next-Basket Recommendation

Next-basket recommendation has been studied in different domains. In the field of e-commerce, the next-basket recommendation is an important part of many e-commerce websites [7] proposes a traditional model that mixes Markov chains and factorization [4] proposes a dynamic recurrent basket model based on RNN and uses max pooling to get the set embedding [8] proposes an encoder-decoder framework that uses average pooling to get set embedding and uses attention mechanism to apply information from different input sets to different output sets. The maximum pooling method causes information about auxiliary medical activities to be discarded. Information about important medical activities is not emphasized in the average pooling approach. Based on the limitations of both of them, we propose a set embedding representation based on a soft-attention mechanism to avoid the above-given information loss problem [5] obtains set embedding by constructing a heterogeneous graph that considers semantic relationships between sets, items, users, and categories. DNA sequences in the biological field are a kind of sequence data [9, 10] carry out effective research in DNA sequence patterns. However, in the medical field, similar problems have been rarely studied [3] handle high-dimensional input vectors by linear dimensionality reduction and predicts the diagnosis of the next admission based on RNN [11] predicts the next clinical event based on LSTM and attention mechanisms. Both deal only with structured information, i.e., medical activities or diagnostic results and do not make use of unstructured information, i.e., medical history texts. It is undeniable that medical history information has a profound impact on the design of subsequent healthcare strategies. In addition, RNN-based models process sequential data in a serial manner. This inevitably results in slow computation speed. The serialized computation only utilizes the temporal information of the sequence of hospitalization days and ignores the interactions among hospitalization days.

### 2.2. Attention Mechanism

The attention mechanism is a feature extraction method. Before it was proposed there were also other feature extraction methods such as Hidden Markov Models [12] and Genetic Algorithms [13] applied in the field of gesture recognition. From a conceptual perspective, the attention mechanism can selectively filter out a small but important amount of information from the vast information but the filtered ones are important and focus attention on them while ignoring the unimportant information. The implementation is done by training to assign different weight coefficients to each message, and then weighting and summing them to obtain the overall representation. The attention mechanism is an essential concept in neural networks. With the introduction of Transformer [14], the self-attention mechanism is widely used. and even outperformed CNN and RNN on many vision related tasks [15] and language related tasks [16]. Transformer-based variants also achieve great success in the field of text processing [17, 18]. Self-attention mechanism also achieves advanced performance in recommendation systems [19, 20]. Compared with RNN and LSTM that specialize in sequence data, self-attention is more likely to capture long-term dependency in sequences and facilitate parallel computation.

### 2.3. Generative Adversarial Network

A generative adversarial network is a machine learning framework consisting of two neural networks [21]. It is implemented as two networks competing against each other, one of which is a generator network that captures features of real sample data to generate fake data. The other is the discriminator network, which observes both real and fake data to discriminate the authenticity of the input. The application of generative adversarial networks showed great success in image generation research [22]. Although there are applications in the field of recommendation systems [23, 24], the application of adversarial learning in temporal set recommendation is an unexplored task. Inspired by the application of generative adversarial networks in image multi-tag recommendation [6], we introduce generative adversarial networks into our study.

## 3. Preliminaries

### 3.1. Data Description and Preprocessing

The EMR dataset used in this study comes from the electronic medical record database of a top-notch hospital. As shown in Figure 1, each medical record contains the following information:

- Medical history. The medical history is textual data which includes the patient's past history, current medical history, and allergy history
- Medical activity. This information includes daily medical activities such as medications, biochemical tests, etc

In our collected dataset, according to the hospital's EMRs system, we regarded a patient's admission process as an EMR record.  Table 1 shows the demographics of patients in the dataset. From the table, firstly we can discover that all breast cancer patients are female patients. Secondly, patients are mainly centered in the aged of 40–70 years, and most patients are from rural areas. Finally, the vast majority of patients are negative for HCV, and many patients did not have previous CT or MRI examinations.

In order to integrate and utilize the above-given data, we conduct the following preprocessing steps. Firstly, inspired by [25], past history, current medical history, and allergy history are combined and meaningless characters are removed. Secondly, removing duplicate activities and unify English and Chinese names for medical activities. Thirdly, records with too few or too many days of inpatient stay are removed. Finally, the records are truncated with 70% to 80% of inpatient days and medical activities that occurred on the last day after interception are regarded as real next-day medical activities since the purpose of our study is not to recommend medical activities for the last day of hospitalization.  Table 2 shows more detailed statistics of our data.

### 3.2. Problem Formalization

Formally, we define all the unique inpatients and medical activities in the entire dataset as *𝕌*={*u*_1_, *u*_2_,…*u*_*N*_} and *𝕍*={*v*_1_, *v*_2_,…*v*_*M*_} with size N and *M,* respectively. And, let *𝕋*={*t*_1_, *t*_2_,…*t*_*N*_} be the set of medical histories, with each *t*_*i*_ corresponding to *u*_*i*_. *𝕎*={*w*_1_, *w*_2_,…*w*_*J*_} is a lexicon of words that appeared in medical histories, and each *t*_*i*_ is an indefinitely long sequence of multiple *w*, *t*_*i*_=(*w*_*i*,1_, *w*_*i*,2_,…*w*_*i*,*j*_). For inpatient *u*_*i*_, using a sequence of embedding to record the inpatient days *D*_*i*_=(*d*_*i*,1_, *d*_*i*,2_,…*d*_*i*,*k*_), where *d*_*i*,*k*_ is the inpatient day embedding that is formalized by a function *f* : *𝒫*(*𝒱*)⟶*ℝ*^*d*_*e*^. *f* is a mapping from the set of medical activities that occurred in a day to a vector of fixed size *d*_*e*, where *𝒱*⊆*𝕍* is a set containing the medical activities which occurred on that day. The goal of our study can be formalized as follows:

(1) $$\begin{array}{c} V_{i,k+1}=f_{rec}\left(d_{i,1},d_{i,2},\ldots d_{i,k},t_{i},W\right)\text{,} \end{array}$$

where **W** are learned parameters, *𝒱*_*i*,*k*+1_ is the set of next-day medical activities recommended by the model.

This problem can be formalized as a supervised learning task, which first trains a recommendation model based on a large number of historical records (including medical history and medical activities since admission) and then recommends the sets of medical activities for the next-day based on the trained model. If the input is only medical activities, then all the model learns is the treatment pattern without personalized information. For this, we conduct joint learning of medical history to address this aspect of personalization. The key idea is to learn to focus on personalized information, which is patient-specific. The joint optimization of the proposed recommendation network simultaneously allows to learn aspects of personalization.

## 4. Proposed Method

The framework of the proposed NDMARec is shown in Figure 2, which consists of four parts: inpatient day embedding, encoder based on multihead self-attention, generative adversarial network, and fusion module.

The first inpatient day embedding is motivated by the medical commonsense that the medical activities that occur during hospitalization differ in importance from one another. Therefore, the concept of inpatient day embedding is proposed, which is obtained by dynamically weighting the included medical activities. Specifically, by training the model to assign different weight coefficients to different medical activities for enhancing the information of important medical activities while suppressing but not discarding the information of ancillary medical activities. This approach we propose effectively deals with the information loss problem [4, 8] caused. The second component inspired by [14] learns potential information between inpatient days and medical history through multihead self-attention, and this component takes inpatient day embedding and word embedding as input. It effectively deals with the limitations caused by RNN-based models [4, 5, 8]. The self-attention module introduces position encoding into the inpatient day vector as temporal information. The self-attention mechanism captures the interactions between inpatient days. This module implements parallel processing by matrix multiplication to speed up the computation. The detailed rationale is in Section 4.2.2. The third part consists of a generator and a discriminator, which generate medical activities based on hidden features and discriminate true and false, respectively. The fourth component is the fusion of potential features learned by the second component to achieve personalization.

### 4.1. Inpatient Day Embedding

A key issue of next-day medical activities recommendation is how to represent medical activities occurred on a day as a vector. That is, the vector length should not be too long and the distribution should not be too sparse. Try to represent as much information as possible with a dense short vector, while paying attention to the importance of different medical activities within the same day, i.e., the influence on subsequent medical activities. Most existing studies use a M-dimensional one-hot vector **s**=[*s*_1_, *s*_2_,…, *s*_*M*_] to solve this, where *s*_*j*_=1, if *v*_*j*_ ∈ *𝒱*; *s*_*j*_=0, otherwise. This type of representation has two drawbacks: (1) the dimension of **s** is too large while active elements are sparse; (2) the importance of different medical activities is not considered.

To overcome above issues, an embedding method based on soft-attention is designed. Association rule analysis shows that certain medical activities always occur within the same day due to the synergy between them [26]. Based on this, we propose to use word embedding that learns a dense vector with small dimension for each medical activity. Formally, let **W**_*e*_ ∈ *ℝ*^*d*_*e*×*M*^ denote the embedding matrix for medical activitiy, where *d*_*e* is the embedding dimension. Each medical activity is encoded as a one-hot column vector **v** ∈ *ℝ*^*M*^, where *v*_*i*_-th value is 1 and other values are zeros. Then, **e**=**W**_*e*_**v** denotes the embedding vector for medical activity *v*. It is well known that embedding can encode objects with low-dimensional vectors and still preserve their meaning [27]. Considering the different importance of medical activities occurred on a day, they should be treated differently to enhance the information of important medical activities and avoid losing the information of auxiliary medical activities. Therefore, the proposed embedding method is formalized as follows:

(2) $$\begin{array}{c} d_{k}=\overset{n_{k}}{\underset{i=1}{\sum }}\alpha_{i}e_{i}\text{,}\\ \alpha_{i}=q^{⊤}\sigma \left(W_{v2\;d}e_{i}+b\right)\text{,} \end{array}$$

where trainable parameters **q** ∈ *ℝ*^*d*_*e*^, **b** ∈ *ℝ*^*d*_*e*^ and **W**_*v*2 *d*_ ∈ *ℝ*^*d*_*e*×*d*_*e*^ control weights, *α*_*i*_ is the attention weight corresponding to the medical activity *v*_*i*_.

### 4.2. Encoder Based-on Multihead Self-Attention

RNN is the most commonly used model for temporal data mining, which usually processes the sequence data in order. The existing solutions to problems similar to our study are mostly based on RNN. or its variants such as LSTM and GRU. But none of them completely solve the issues of long-term dependency. This also means that the RNN-based network structure may not take full advantage of some of the medical activities at the time of the patient's initial admission thus reducing the model performance. As a result, in this study, multihead self-attention is applied to inpatient day sequences and medical histories because it focuses on each inpatient day or word simultaneously, which not only improves the parallelism but also alleviates long-term dependency. Multiple attention heads enable the network to capture richer information. For the inpatient day and the medical history, using two neural networks with the same structure to process them separately. The difference between the two is only in the way the final information is aggregated. As shown in Figure 1, one uses attention-based aggregation while the other uses average aggregation. Next, the structure of the encoder based on multihead self-attention will be described in detail.

#### 4.2.1. Position Encoding

To exploit the temporality between inpatient days and the sequentiality of words in the medical history, position encoding is set for inpatient day embedding and word embedding to represent relative positions, respectively.

(3) $$\begin{array}{c} \left\{\begin{array}{c} PE\left(pos,2i\right)=\sin\left(\frac{pos}{100^{\left(2i/d\_e\right)}}\right)\text{,}\\ PE\left(pos,2i+1\right)=\cos\left(\frac{pos}{100^{\left(2i/d\_e\right)}}\right)\text{,} \end{array}\right) \end{array}$$

where pos ∈ (0, *n*_*u*_] and *i* ∈ [0, *d*_*e*/2] denote position and dimension, respectively. For the sequence of inpatient days, pos denotes the pos-th day since admission and *n*_*u*_ denotes the number of inpatient days up to the present. For medical history, pos and *n*_*u*_ denote the position of the word in the text and the number of words contained in the text, respectively. With the *PE*(·) function, the contextual information of different positions is calculated. Afterwards, as shown in Equation (4), the inpatient day embedding and word embedding are summed with their position encoding respectively as the input to the downstream task.

(4) $$\begin{array}{c} \left\{\begin{array}{c} x_{i}^{d}=d_{i}+PE\left(i\right)\text{,}\\ x_{j}^{w}=w_{j}+PE\left(j\right)\text{,} \end{array}\right) \end{array}$$

where **x**_*i*_^*d*^ and **x**_*j*_^*w*^ are the inputs for the encoder used to process inpatient days and medical history, respectively.

#### 4.2.2. Multihead Self-Attention and Residual Connection

Figure 3 shows the detailed structure of the self-attention mechanism. The left and right of Figure 3 indicate the input vector processed by Equation (4) and the output vector processed by the self-attention mechanism, respectively. The inpatient day embedding and the word embedding after adding the position encoding are translated as **q**, **k**, and **v** through the three mapping matrices (**W**_*Q*_, **W**_*K*_, and **W**_*V*_) of their modules, respectively.

(5) $$\begin{array}{c} \left\{\begin{array}{c} q=W_{Q}x+b_{Q}\text{,}\\ k=W_{K}x+b_{K}\text{,}\\ v=W_{V}x+b_{V}\text{,} \end{array}\right) \end{array}$$

where **W**_*Q*_, **W**_*K*_ and **W**_*V*_ ∈ *ℝ*^*d*_*e*×*d*_*k*^ denote the mapping matrices applied to the inpatient day embedding or the word embedding, respectively. **b**_*Q*_, **b**_*K*_ and **b**_*V*_ ∈ *ℝ*^*d*_*k*^ denote the bias, respectively.

Each **q** is multiplied by a matrix **K** concatenated by the transpose of all **k** of the whole sequence and then processed by softmax to obtain its self-attention weights for the elements at other positions of this sequence. This is then multiplied by all **v** and summed to obtain the output at the current position.

(6) $$\begin{array}{c} Attention\left(q,K,V\right)=softmax\left(\frac{qK^{⊤}}{\sqrt{d}}\right)V\text{.} \end{array}$$

Compared with RNN, the self-attention mechanism focuses on the whole sequence simultaneously, which ensures parallel computation to reduce the time complexity of the algorithm. We compute the output of all elements of the entire sequence simultaneously by concatenating the query vectors as a matrix **Q** to achieve parallel computation:

(7) $$\begin{array}{c} Attention\left(Q,K,V\right)=softmax\left(\frac{QK^{⊤}}{\sqrt{d}}\right)V\text{,} \end{array}$$

where $\left(1/\sqrt{d}\right)$ is the scaling factor used to alleviate the gradient vanishing. Multiple attention heads are used to capture richer information and features and the learned features are combined as output:

(8) $$\begin{array}{c} A=MultiHead\left(Q,K,V\right)=Concat\left(H_{1},H_{2},\ldots ,H_{h}\right)W_{o}\text{,} \end{array}$$

where *H*_*i*_=Attention(**Q**, **K**, **V**) and **W**_*o*_ ∈ *ℝ*^*h*·*d*_*k*×*d*_*e*^, *h* denotes the number of self-attention heads, Concat (·) is a vector concatenation operation.

As shown in Figure 2, referencing most network structures, the residual connection [28] and layer normalization [29] are also applied to our model. The purpose of layer normalization is to normalize the state of the hidden layer in the neural network to a standard normal distribution to accelerate convergence. The residual connection is essentially an additive node. It is responsible for passing the upper gradient to the lower level in back propagation to preserve the original state of the gradient, which reduces the risk of gradient disappearance and gradient explosion in the network and makes the whole network more active in the learning state.

(9) $$\begin{array}{c} h=Layer\;Norm\left(A+FFN\left(A\right)\right)\text{,} \end{array}$$

(10) $$\begin{array}{c} FFN\left(A\right)=W_{F2}\left(ReLU\left(W_{F1}A+b_{F1}\right)+b_{F2}\right)\text{,} \end{array}$$

where **W**_*F*1_ ∈ *ℝ*^*d*_*e*×*d*_*f*^ and **W**_*F*2_ ∈ *ℝ*^*d*_*f*×*d*_*e*^ are trainable parameters, ReLU (·) is the activation function. **h** is the hidden vector.

#### 4.2.3. Attention-Based Aggregation of Inpatient Day Information

There is time-dependency between next-day medical activities and previously occurring medical activities. Specifically, we consider that different sequences of inpatient days may have different effects on different next-day medical activities. For example, if an inpatient suffers adverse reaction to an injectable drug, the patient's subsequent medical activities will be altered as a result. In addition to the need to change the medication, measures need to be taken to mitigate the adverse reaction to ensure smooth followup treatment. As mentioned previously, the impact of medical activities that occurred previously is different. In addition, the medical activities that occurred on the last day are more influential. Hence, designing an attention module to focus on previous inpatient days and leverage their different impact.

(11) $$\begin{array}{c} z^{d}=\overset{K}{\underset{k=1}{\sum }}\frac{e_{kK}}{\sum_{i}^{K}e_{iK}}h_{k}^{d}\text{,} \end{array}$$

where **e**_*iK*_=MLP(Concat(**h**_*i*_, **h**_*K*_)). MLP is a multilayer perceptron and **h**_*k*_^*d*^ and **h**_*i*_ are the hidden vectors calculated from Equation (9). *K* is the number of days since admission.

#### 4.2.4. Medical History Information Aggregation

Personalization is an important feature of recommendation systems [30]. For this study, the emphasis of personalization is that the model recommends next-day activities that are specific to the patient's condition, rather than simply learning a generic treatment model. Hence, the model incorporates medical history information in its recommendations to improve performance. We adopt an averaging pooling strategy to aggregate the hidden states of words in the medical history learned by the multi-head self-attention in Section 4.2.2.

(12) $$\begin{array}{c} z^{w}=\frac{1}{J}\overset{J}{\underset{j=1}{\sum }}h_{j}^{w} \end{array}$$

where *J* indicates the number of self-attended heads in Section 4.2.2.

### 4.3. Generating Adversarial Network

In this study, we propose to explore adversarial learning for next-day medical activity recommendations. The idea is to use the additional adversarial loss for medical activity prediction, thus ensuring that the recommended medical activities have a distribution similar to the ground truth. Specifically, if the recommended results are not similar to the actual distribution of the ground truth, the adversarial loss is introduced to penalize the recommendation network.

The loss of generator *𝒢* and discriminator *𝒟* are incorporated into our model separately, where the medical activities from the generator network are considered as generated labels. And, there is a discriminator to distinguish the generated labels from the ground truth labels, that is, the real next-day medical activities. The purpose of *𝒢* is to fool *𝒟* by generating medical activities that resemble real activities occurred on next-day, which is achieved by minimizing the following loss function:

(13) $$\begin{array}{c} L_{G}=\frac{1}{N}\overset{N}{\underset{i=1}{\sum }}\left[\log\;\left(1-D\left(G\left(z_{i}^{d}\right)\right)\right)\right]\text{,} \end{array}$$

Where *ℒ*_*𝒢*_ denotes the generator loss and **z**_*i*_^*d*^ is the output of Section 4.2.3, which is the inpatient day information used for next-day medical activity recommendations. The *𝒢* predicts generalized medical activity **V**_*G*_. It consists of two linear layers, followed by a fully connected layer for prediction. And, there is also a cross-entropy loss function:

(14) $$\begin{array}{c} L^{\left(g\right)}=-\frac{1}{M}\overset{M}{\underset{i=1}{\sum }}p_{i}\log{\hat{p}}_{i}+\left(1-p_{i}\right)\log\;\left(1-{\hat{p}}_{i}\right)\text{,} \end{array}$$

where *p*_*i*_ indicates whether a medical activity occurred on next-day and ${\hat{p}}_{i}$ is a medical activity predicted by *𝒢*.

The task of *𝒟* is to distinguish whether the input is generated or ground truth. If the *𝒟* can distinguish between ground truth and recommendation results, the recommendation network is penalized. It is trained by the following equation:

(15) $$\begin{array}{c} L_{D}=-\frac{1}{N}\overset{N}{\underset{i=1}{\sum }}\left[\log\;\left(D\left(V_{Ti}\right)\right)+\log\;\left(1-D\left(V_{Gi}\right)\right)\right]\text{,} \end{array}$$

where **V**_*Ti*_ is a set of medical activities occurred on the next day. The *𝒟* consists of two linear layers with ReLU and uses the sigmoid activation function at the end.

### 4.4. Information Fusion

Long-term orders exist in the clinical record, which occur daily and are not affected by changes in the patient's condition. For example, diabetic diet, blood pressure measurement, etc. To retain such long-term orders, a frequency statistical component is designed to simulate them. Specifically, the medical activities that have occurred since admission are recorded by a vector **L**^*p*^=[*l*_1_^*p*^, *l*_2_^*p*^,…, *l*_*M*_^*p*^], where *l*_*j*_^*p*^(*j* ∈ [1, *M*]) denotes the number of medical activity *v*_*j*_ has occurred.

As previously illustrated, our study extracted information about the patient's medical history in addition to considering medical activity in the recommendation process. This is work that has not been done by most studies about temporal set prediction and next-basket recommendation [31] that focus more on sequential patterns. Inspired by [32], this study integrates the personalized information of medical history with the sequential pattern of medical activities to generate the final recommendation results. Notably, our study employs an additive fusion strategy controlled by hyperparameters, which eliminates a large amount of multiplicative computations in fusing features to speed up the computation and achieve competitive results compared to the concatenation method. Therefore, the final recommended results for next-day medical activities are represented as follows:

(16) $$\begin{array}{c} \hat{y}=\sigma \left(\left(1-\alpha ⊙\beta \right)⊙\left(W_{d}z^{d}+b_{d}\right)+\alpha ⊙l^{p}+\lambda \left(W_{txt}z^{w}+b_{txt}\right)\right)\text{,} \end{array}$$

where **W**_*d*_ and **W**_*txt*_ ∈ *ℝ*^*d*_*e*×*M*^ are learnable parameters, 1 ∈ *ℝ*^*m*×1^ is an all-one vector, ⊙ denotes elementwise Hadamard product, *λ* is a hyperparameter, *β* ∈ *ℝ*^*M*×1^ is a vector composed of 0 or 1 and 1 means the corresponding dimension of **l**^*p*^ is nonzero, respectively. *α* is a weight factor used to balance the information from long-term orders and learned. The *α* is calculated as follows:

(17) $$\begin{array}{c} \alpha =\sigma \left(W_{p}l^{p}+b_{p}\right)\text{.} \end{array}$$

### 4.5. Loss Function

We build an end-to-end model to jointly train the above parts and choose Mean Square Error (MSE) as a loss function. The objective function to be minimized is defined as follows:

(18) $$\begin{array}{c} L=\frac{1}{N}\sum {\left(y-\hat{y}\right)}^{2}+\gamma L^{\left(g\right)}\text{,} \end{array}$$

where ***y*** and $\hat{y}$ denote the ground truth and recommended next-day medical activities, respectively. *γ* is a hyperparameter.

## 5. Experiments

In this section, we conduct extensive experiments to validate the effectiveness of the proposed method. We first the evaluation metrics and the comparison baseline. Then, the performance comparison of our method with classical and state-of-the-art methods is given. Finally, the effectiveness of each module of our method is verified by the ablation study, and the interpretability of the model is discussed by visualizing the attention coefficient during inpatient day embedding generation and the attention coefficient during next-day medical activity recommendation.

### 5.1. Experimental Settings

We omit the dataset description since it has been introduced in Section 3.1. Other experimental settings will be described in the following parts.

#### 5.1.1. Evaluation Metrics

There is a ranking list of top-K items generated from the output and the *K* is set to 10, 15, 20, and 25, respectively. We use Recall and NDCG to evaluate our method. Next-day medical activities recommendation can be regarded as a special kind of multilabel classification problem.

(i) Recall is a widely used measure for multi-label classification [33]. For each patient, recall is calculated as follows:
  (19) $$\begin{array}{c} Recall@K\left(u_{i}\right)=\frac{\left|{\hat{S}}_{i}\cap S_{i}\right|}{\left|S_{i}\right|}\text{.} \end{array}$$
(ii) NDCG is a measure that considers the ranking order of recommendation results [34]. For each patient, NDCG is calculated as follows:
  (20) $$\begin{array}{c} NDCG@K\left(u_{i}\right)=\frac{\sum_{k=1}^{K}\delta \left({\hat{S}}_{i}^{k},S_{i}\right)/\log_{2}\;\left(k+1\right)}{\sum_{k=1}^{\min\;\left(K,\left|S_{i}\right|\right)}1/\log_{2}\;\left(k+1\right)}\delta \left(v,S\right)=\left\{\begin{array}{cc} 1\text{,} & v\in S\text{,}\\ 0\text{,} & v\notin S\text{.} \end{array}\right) \end{array}$$

We adopt the average recall and NDCG of all inpatients as metrics.

#### 5.1.2. Compared Methods

We compare our method with the following baselines, including both classical and the state-of-the-art methods:

- PersonalTOP: it counts the medical activities that have occurred since admission for different inpatients and then makes recommendations.
- ItemTransfer: it first constructs a transmission relationship (represented by an adjacency matrix) between medical activities between different hospitalization days since the admission of a given patient and then recommends medical activities for the next day in conjunction with the medical activities of the last day.
- DREAM [4]: it is an earlier method of using deep neural networks for next-basket recommendations. DREAM uses max pooling to generate basket's embedding and uses RNN to generate recommendation results.
- Sets2sets [8]: it uses average pooling to generate set embedding and designs a GRU-based encoder-decoder framework for multi-period prediction.
- DHNTSP [5]: it is the state-of-the-art method in temporal set prediction based on LSTM, which designs a set representation method based on a heterogeneous information network.

#### 5.1.3. Configuration of Our Method

We divide our dataset into train, validation, and test set across inpatients with ratios of 70%, 10%, and 20% to do experiments. PyTorch is used to build our model and Adam [35] is adopted as the optimizer. The stacked layers of self-attention is applied to the inpatient day sequence and medical history of 1 and 2, respectively. The dimension of the embedding, *d*_*e*, is set to 32. The hyperparameters *λ* and *γ* are both set to 0.5.

### 5.2. Performance Analysis

To demonstrate the effectiveness of our next-day medical activities recommendation model, we compared NDMARec with all comparison methods. The results are shown in Table 3 and Figure 4. And, the proposed NDMARec model achieved better performance in most cases. In addition, there are some interesting findings in these comparison experiments.

Firstly, PersonalTOP achieves better performance. This is because many medical activities are long-term medical orders in our dataset, which means their frequency will be high. So even though PersonalTOP does not consider the time dependency, it achieves comparable performance.

Secondly, ItemTransfer achieves better performance than PersonalTOP because it considers the transfer relationships of medical activities between adjacent inpatient days. This shows that capturing the transfer relationships between medical activities can improve performance.

Thirdly, although DREAM and Sets2sets use neural networks to focus on inpatient days, they do not achieve better performance. This is because they do not consider the importance of medical activities when generating inpatient day embedding. The max pooling used by DREAM results in the loss of information about ancillary medical activities, while the average pooling used by Sets2sets lead to information about important medical activities not being highlighted. Sets2sets also introduces an attention mechanism compared to DREAM but does not achieve a significant performance improvement. This is because the objective function of Sets2sets is set to emphasize medical activities which occur less frequently, which may suppress the prediction effect of medical activities that belong to long-term medical orders.

Finally, in most cases, NDMARec outperforms other methods. The previous models did not have a medical history feature extraction module and information fusion module. They only use structured data, i.e., daily medical activity since admission, as input to recommend next-day medical activity. NDMARec, however, uses not only medical activities as input, but also unstructured data, i.e., medical history text, as input. The two features are fused to recommend next-day medical activities. In addition to the import of medical history information, the next section Ablation Study also illustrates the advanced nature of each module of NDMARec. Compared to PersonalTOP and ItemTransfer, NDMARec captures the dynamic temporal dependency of medical activities between inpatient days. The attention mechanism is also used to differentiate the impact of inpatient days. Compared to DREAM, Sets2sets, and DHNTSP, NDMARec alleviates long-term dependency by multihead self-attention that simultaneously focus on each day's medical activities. In addition, an embedding method based on soft-attention is adopted to balance the importance of different medical activities when designing inpatient day embedding and the use of generative adversarial networks allows our network to learn features that are more conducive to recommending accurate medical activities, both of which result in better performance of our method.

### 5.3. Ablation Study

To verify the effect of the components of our model, we design the following simplified variant of our model:

- NDMARec-MP: it takes the max value of each dimension of the medical activity embedding in the inpatient day embedding component imitating DREAM, which loses a lot of information
- NDMARec-AP: it takes average pooling for medical activity embedding to get inpatient day embedding, which causes important medical activities not being highlighted
- NDMARec-NH: it removes the component that handles medical history which means that the effect of medical history is not considered
- NDMARec-NA: it removes the generative adversarial network during training
- NDMARec-A-B: A and B denote the number of self-attention stacking layers applied to the inpatient days and medical history, respectively

The results of the ablation study are shown in Table 4 and Figure 5. From the results, we can draw the following conclusions: firstly, the inpatient day embedding method based on the soft-attention outperforms average pooling and max pooling, which indicates that our embedding method selects more important medical activities adaptively. Secondly, the fusion of medical history significantly improves performance. Observations indicate that fusing medical history to assist medical activities implementation can increase the personalization of recommendation results and improve the performance. Thirdly, the use of generative adversarial networks in the training phase improves the learning ability of the model. This shows that the joint use of generators and discriminators can help our model learn effective features, which could improve the generalization ability of the recommendation network by penalizing it. Finally, we explore the effect of the number of self-attention stacking layers. Surprisingly, the model performance does not improve with increasing the number of layers. Observations indicate that the best performance is achieved when setting the number of self-attentive layers handling inpatient days and medical history to 1 and 2, respectively. This may be due to the fact that the dependency relations of the inpatient day sequences are not as complex as the sentences in the machine translation task and the words in the medical history text are carefully cleaned and preprocessed. Therefore, a smaller number of layers is sufficient to obtain good performance while too many layers could lead to overfitting. Similar observations can be found in [36].

### 5.4. Visualization and Interpretability

To discuss the interpretability of our method, we randomly selected a sample for which the daily medical activities are shown in Table 5. The corresponding attention coefficients for this sample during the generation of inpatient day embedding and during the recommendation of next-day medical activities are visualized as shown in Figure 6. The red part represents medical activities that occurred during the day, the green part represents inpatient days, and the bottom arrow denotes the sequence order of inpatient days. The lightness of red indicates the importance of the medical activity for that day, and the lightness of green denotes the influence of this day on the recommendation of the medical activities for the next-day.

From Table 5 and Figure 6, it is easy to observe that our model does focus attention on certain important medical activities, which means that when generating the inpatient day embedding, the attention mechanism adaptively enhances certain important medical activities (e.g., Matrine and sodium chloride injection on the 4-th day and Pantoprazole sodium for injection and Cisplatin injection on the 7-th day) and suppressing the features of ancillary medical activities (e.g., Common food, Tertiary care on the 2-nd day). This attention mechanism is clearly consistent with medical theory and demonstrates the validity and interpretability of the inpatient day embedding module. The distribution of attention when recommending next-day medical activities also matches the design goals of this study. The bottom left corner of Figure 6 indicates that the recommendation model based on multihead self-attention does not suffer from the remote dependence issue of the RNN-based model; that is, our model does not ignore the medical activity that occurs when the patient is first admitted to the hospital, and not only that, our model assigns a relatively high attention coefficient to it, which indicates that the medical activities that occurred on the first day of the patient's admission continue to influence the planning and implementation of subsequent treatment strategies.

The visualization also revealed the interesting phenomenon that the higher the number of medical activities occurring on a given day does not indicate a greater contribution of that day to the recommendation of medical activities on the following day. This is also true in actual clinical care. A cancer patient may only take oral anticancer drugs on a certain day, but the subsequent medical activities must be arranged and formulated around alleviating the side effects of that drugs, which means that the day the oral anticancer drugs are taken has a significant impact on the subsequent medical activities, and the attention coefficient allocated to that day becomes correspondingly larger. The significantly larger attention coefficient assigned for the current last day demonstrates that our method focuses on the influence of the patient's current day's medical activities when recommending next-day medical activities. This is in line with the idea of considering the user's current interests in session-based recommendations [37, 38]. However, most studies in session-based recommendation explicitly combine current interests with long-term user preferences; our method relies entirely on a self-attention mechanism to make the model autonomously emphasize current information, which illustrates that our recommendation model can automatically discover the importance of the current inpatient day.

## 6. Conclusion

In this paper, we propose a new end-to-end model (called NDMARec) to recommend next-day medical activities for inpatients based on medical history and occurred medical activities. NDMARec extracts dependencies between different inpatient days and fuses medical histories for recommendations. Features of medical activities and medical histories are learned by an encoder based on a multihead self-attention. In addition, we incorporate a generative adversarial network to enhance the learning capability of the model during the training phase. The results of multiple comparative experiments and ablation study demonstrate the better performance of our model and the effectiveness of each module.

Current research in the area of medical activity recommendation is relatively small. The main constraints are the difficulty in obtaining real data, the complexity of the data, and the diversity of real clinical scenarios. There is also a lot of unused information for our study such as patient survival and readmission rates. In the future, we will consider including patient survival and readmission rates when recommending next-day medical activities to further suggest the accuracy and validity of the recommended outcomes. In addition, we will also deepen cooperation with hospitals to train different recommendation models for different diseases to enhance the personalization of recommendation results.

## Figures and Tables

**Figure 1:** An example of a medical record in a dataset.

**Figure 2:** Framework of the proposed model.

**Figure 3:** The detailed process of self-attention.

**Figure 4:** Results comparison on our dataset, where *K* changes from 10 to 25 with a step size of 5.

**Figure 5:** Ablation study of NDMARec.

**Figure 6:** Visualization of the attention coefficient.

**Table 1:** The demographics of patients.

Demographics	Collected EMRs dataset in 811 patients
Gender distribution	Female: 811 (100%); male: 0 (0%)
Age distribution	0∼40: 110 (13.5%); 40∼70: 663 (81.8%); 70+: 38 (4.7%)
Region distribution	Rural: 496 (61.2%); Urban: 315 (38.8%)
HCV distribution	N: 774 (95.4%); P: 37 (4.6%)
CT/MRI previous	Yes: 97 (12%); No: 714 (88%)

**Table 2:** Statistics of our dataset.

Description	Number
The number of records	10941
The number of medical activities	3204
Mean number of inpatient days	9
Mean number of medical activities per day	8
Mean number of words in the medical history	168

**Table 3:** Performance comparison of all methods (%). The best performance and the second best performance are shown in bold and italic font, respectively.

Method	Recall@10	NDCG@10	Recall@15	NDCG@15	Recall@20	NDCG@20	Recall@25	NDCG@25
PersonalTop	84.02	88.81	86.60	88.80	87.76	89.09	88.69	89.43
ItemTransfer	85.45	89.99	88.48	90.19	89.55	90.42	90.06	90.56
DREAM	73.20	78.88	77.89	79.99	80.93	81.18	83.24	82.16
Sets2sets	77.74	79.85	82.33	80.86	84.98	81.83	86.68	82.54
DHNTSP	**88.20**	*92.98*	*91.83*	*93.40*	*93.12*	*93.69*	*93.97*	*93.96*
NDMARec	*88.19*	**93.92**	**92.14**	**93.90**	**93.71**	**94.08**	**94.62**	**94.23**

**Table 4:** Results of ablation study (%).

Model	Recall		NDCG	
	@10	@20	@10	@20
NDMARec-MP	86.71	89.58	91.11	90.09
NDMARec-AP	88.08	90.65	93.24	91.48
NDMARec-NH	86.78	90.09	91.23	90.58
NDMARec-NA	87.01	92.44	92.05	93.01
NDMARec-6-6	86.36	89.09	90.96	89.73
NDMARec-3-3	81.01	89.92	91.92	90.69
NDMARec	**88.19**	**93.92**	**93.71**	**94.08**

**Table 5:** Order of inpatient days and medical activities that occurred on that day.

1	2
Peripheral blood routine	0.9% sodium chloride injection
Routine ECG examination	L-carnitine injection
Tertiary care	Tertiary care
Common food	Common food
Liver function	Matrine and sodium chloride injection
Renal function	
CA15-3	
Blood sugar	
Carcinoembryonic antigen assay (CEA)	

3	4
0.9% sodium chloride injection	0.9% sodium chloride injection
L-carnitine injection	L-carnitine injection
Matrine and sodium chloride injection	Common food
Tertiary care	Tertiary care
Common food	Matrine and sodium chloride injection
Central venous catheterization	Nursing care of arteriovenous catheterization
Lidocaine hydrochloride injection	Tube sealing after 15 ml saline infusion
Heparin sodium injection	
Nursing care of arteriovenous catheterization	
Tube sealing after 15 ml saline infusion	
Dexamethasone acetate tablets	

5	6
0.9% sodium chloride injection	Paclitaxel injection
L-carnitine injection	L-carnitine injection
Common food	Matrine and sodium chloride injection
Tertiary care	Tropisetron hydrochloride for injection
Matrine and sodium chloride injection	Pantoprazole sodium for injection
Nursing care of arteriovenous catheterization	5% glucose injection
Tube sealing after 15 ml saline infusion	ECG monitoring
Adhesive tape for indwelling needle	Blood oxygen saturation monitoring
	Dexamethasone sodium phosphate injection
	Promethazine injection
	Tertiary care
	Common food
	Sodium deoxynucleotide injection
	0.9% sodium chloride injection
	Nursing care of arteriovenous catheterization
	Tube sealing after 15 ml saline infusion
	Adhesive tape for indwelling needle

7	8
Tropisetron hydrochloride for injection	0.9% sodium chloride injection
L-carnitine injection	L-carnitine injection
Matrine and sodium chloride injection	Matrine and sodium chloride injection
0.9% sodium chloride injection	Tropisetron hydrochloride for injection
Blood oxygen saturation monitoring	Pantoprazole sodium for injection
5% glucose injection	5% glucose injection
ECG monitoring	ECG monitoring
Pantoprazole sodium for injection	Blood oxygen saturation monitoring
Cisplatin injection	Pidotimod oral liquid
Common food	Compound zaofan pill
Sodium deoxynucleotide injection	Peripheral blood routine
Tertiary care	Tertiary care
Nursing care of arteriovenous catheterization	Common food
Tube sealing after 15 ml saline infusion	Sodium deoxynucleotide injection
Adhesive tape for indwelling needle	Cisplatin injection
	Nursing care of arteriovenous catheterization
	Tube sealing after 15 ml saline infusion
	Adhesive tape for indwelling needle

## Data Availability

The EMR dataset used in this study was obtained from the electronic medical record database of Liaoning Cancer Hospital in China. Because of patient privacy issues, they are not directly disclosed.
